# Bronchial Wall Measurements in Patients after Lung Transplantation: Evaluation of the Diagnostic Value for the Diagnosis of Bronchiolitis Obliterans Syndrome

**DOI:** 10.1371/journal.pone.0093783

**Published:** 2014-04-08

**Authors:** Sabine Dettmer, Lars Peters, Claudia de Wall, Cornelia Schaefer-Prokop, Michael Schmidt, Gregor Warnecke, Jens Gottlieb, Frank Wacker, Hoen-oh Shin

**Affiliations:** 1 Hannover Medical School, Department of Radiology, Hannover, Germany; 2 Hannover Medical School, Department of Respiratory Medicine, Hannover, Germany; 3 Radiologie, Meander Medisch Centrum, Amersfoort, the Netherlands; 4 Radiologie – DIAG, UMC St Radboud, Nijmegen, the Netherlands; 5 Fraunhofer MEVIS, Bremen, Germany; 6 Hannover Medical School, Department of Thoracic and Cardiovascular Surgery, Hannover, Germany; The Hospital for Sick Children and The University of Toronto, Canada

## Abstract

**Objectives:**

To prospectively evaluate quantitative airway wall measurements of thin-section CT for the diagnosis of Bronchiolitis Obliterans Syndrome (BOS) following lung transplantation.

**Materials and Methods:**

In 141 CT examinations, bronchial wall thickness (WT), the wall area percentage (WA%) calculated as the ratio of the bronchial wall area and the total area (sum of bronchial wall area and bronchial lumen area) and the difference of the WT on inspiration and expiration (WTdiff) were automatically measured in different bronchial generations. The measurements were correlated with the lung function parameters. WT and WA% in CT examinations of patients with (n = 25) and without (n = 116) BOS, were compared using the unpaired t-test and univariate analysis of variance, while also considering the differing lung volumes.

**Results:**

Measurements could be performed in 2,978 bronchial generations. WT, WA%, and WTdiff did not correlate with the lung function parameters (r<0.5). The WA% on inspiration was significantly greater in patients with BOS than in patients without BOS, even when considering the dependency of the lung volume on the measurements. WT on inspiration and expiration and WA% on expiration did not show significant differences between the groups.

**Conclusion:**

WA% on inspiration was significantly greater in patients with than in those without BOS. However, WA% measurements were significantly dependent on lung volume and showed a high variability, thus not allowing the sole use of bronchial wall measurements to differentiate patients with from those without BOS.

## Introduction

Bronchiolitis obliterans syndrome (BOS) is the primary long-term complication following lung transplantation and it considerably influences the prognosis of transplant patients [1]. BOS affects up to 60% of lung transplant recipients during the five years following surgery [2]. Histopathologically, bronchiolitis obliterans (BO) is a fibroproliferative process of the small airways and results in multifocal obliteration of the terminal bronchioli [3]. Characteristic histopathology features are a patchy, submucosal fibrosis in the respiratory bronchioles resulting in nearly total or total occlusion of the small airways. The mechanisms by which BO is mediated are manifold and are not yet completely understood. Alloimmune reactivity appears to have a role as well as antibody-mediated rejection, including activation of innate immune cells and response to enviromental and endogenous factors such as infection and aspiration [4].

BO is difficult to quantify histologically due to the nonuniform distribution of fibrosis. Therefore in 1993, a committee of the International Society for Heart and Lung Transplantation (ISHLT) proposed a clinical description of BO, termed bronchiolitis obliterans syndrome (BOS), with a decrease of FEV_1_ (forced expiratory volume in one second) of at least 20% of the postoperative baseline value [5], [6] and unexplained by acute rejection, infection or other complications. The severity of BOS is graded according to the degree of obstruction found in pulmonary function tests (PFT): BOS 1 describes a 20–34% decrease in FEV_1_ from baseline; BOS 2 a 35–49% decrease in FEV_1_; and BOS 3 at least a 50% decrease in FEV_1_ from baseline [6]. Although transbronchial biopsy can be used to establish the diagnosis, it is rarely used because of its low sensitivity [7].

The standard workup for the diagnosis of BOS at our lung transplant center initially includes routine lung function tests, bronchoscopy and CT of the chest. If there are decreased values, especially for FEV_1_, other causes, such as infection, asthma or chronic obstructive disease, are excluded. BOS is diagnosed if no other reason for an obstruction is found and if the impairment persists.

The histopathological changes of the airways seen in BOS result in distinct CT morphological findings such as air trapping [8] and bronchial wall thickening [9] (Figure 1). Other CT findings frequently seen in patients with BOS are bronchiectasis, mucus plugging, and consolidations [9], [10], [11]. However, it has been shown that none of these findings could predict the development of BOS [12]. There have been repeated efforts to use CT findings to diagnose BOS before it results in clinically apparent functional impairment [10], [13]. However, to date these findings have not produced convincing evidence.

**Figure 1:** Typical CT findings of BOS include bronchial wall thickening (A), mosaic attenuation (A), air trapping (B) and bronchiectasis (C).

During the past 10 years, efforts have been made to measure bronchial wall thickness and bronchial lumen [14]. Contemporary software allows automatic segmentation of the bronchial tree and quantification of the bronchial wall and bronchial lumen [15]. Different mathemathical models have been applied with variable accuracy, especially for the smaller and more peripheral airways. The most frequently described method is based on the Full-width-at-half-maximum-principle (FWHM) [16]. However, it has been shown that this method systematically overestimates the wall thickness for small airways [17], [18]. The algorithm used in our study is based on the mathematical integration of Hounsfield intensities (intensity integration) across wall regions [19] as this was found to reduce overestimation of WT in small airways and, therefore, seems especially suited for this particular patient group [20].

Previous studies have shown that bronchial wall thickness quantified on CT data is correlated with the lung function parameters in patients with various airway diseases such as COPD [21], [22], CF [23], and asthma [24], [25].

The purpose of our feasability study is to evaluate whether there is any correlation between the lung function parameters and the CT dimensions of airways and if the airway wall parameters may help to distinguish between lung transplant patients with and those without BOS.

## Materials and Methods

### Prospective Study Design

Written consent was obtained from all of the patients participating in this study. The consent procedure and study were approved by the Ethics Committee of Hannover Medical School (number 5108).

This prospective study was conducted in a single medical center with a large lung transplant program and more than 100 annual lung transplantations [26]. The study is part of a larger research project to develop imaging tools in recipients who develop BOS after lung transplantation so as to allow an earlier diagnosis and more accurate monitoring of the disease process. Our clinical workup in patients following lung transplantation includes routine CT scans performed at six, 12 and 24 months after transplantation. We included all individuals who had undergone double or heart and lung transplantation at our clinic when they were between 18 and 68 years of age and with stable graft function (FEV_1_>90%). Exclusion criteria were severe airway complications after surgery and necessitating intervention, oxygen desaturation during exercise to less than 89% without supplemental oxygen, cardiovascular complications that limited exercise tolerance, single lung and living lobar recipients, and patients with an established diagnosis of BOS at the time of their inclusion and the inability to undergo body plethysmography which may have been due to persistent infection caused by multi-drug-resistant bacteria. Because of the limited number of study patients with clinically manifested BOS during the time between baseline CT and the data inclusion endpoint, we included n = 8, randomly chosen, additional examinations of patients with a clinical diagnosis of BOS for data analysis that fulfilled all of the inclusion criteria stated above with the exception of the availability of a baseline CT with normal PFT.

### Study Participants

Our study patient group consisted of 90 lung-transplant patients. The demographic data are presented in Table 1. There were 53 male patients and 37 female patients with a mean age of 45 years (range 18–65 years) at the time of their examination. For 85 patients it was the first transplantation, and five patients underwent a re-transplantation. Eighty-four patients had a double-lung transplantation, and six patients underwent a heart-lung transplantation; however, none of the patients underwent single-lung transplantation.

**Table 1:** Demographic data of all patients with/without BOS.

		All	Without BOS	With BOS
**Number**	Patients	90		
	Examinations	141	117 (83%)	24 (17%)
**Age (Years)**	At timepoint of CT	45 (18–65)	46 (22–65)	45 (18–66)
**Gender**	Male	53 (59%)	45 (60%)	8 (53%)
	Female	37 (41%)	30 (40%)	7 (47%)
**Transplantation**	Double lung	84 (93%)	70 (93%)	14 (93%)
	Heart-lung	6 (7%)	5 (7%)	1 (7%)
	First transplantation	85 (94%)	72 (96%)	13 (87%)
	Re-transplantation	5 (6%)	3 (4%)	2 (13%)
**Number of CT-examinations**	1	45 (50%)		
	2	40 (44%)		
	3	4 (4%)		
	4	1 (1%)		
**Underlying disease**	Cystic fibrosis	18 (20%)	16 (21%)	2 (13%)
	Emphysema	30 (33%)	26 (35%)	4 (27%)
	Pulmonary fibrosis	20 (22%)	17 (23%)	3 (20%)
	Pulmonary hypertension	5 (6%)	4 (5%)	1 (7%)
	BOS	5 (6%)	3 patients (4%)	2 patients (13%)
	Other	6 (12%)	9 patients (12%)	3 patients (20%)

Of these 90 patients, 45 had one examination, 40 had two examinations, four had three examinations, and one patient had four examinations, resulting in a total of 141 paired CT examinations and lung function tests. One hundred and seventeen examinations were performed in lung transplant patients without BOS and 24 in patients with a clinical diagnosis of BOS (15 were BOS stage 3, two were BOS stage 2, and seven were BOS stage 1). The BOS stages were classified by a pneumologist (CdW) based on FEV_1_ and according to the guidelines of the International Society for Heart and Lung Transplantation (ISHLT) [5]. Other reasons for a reduction of FEV_1_, such as infection, asthma or chronic obstructive pulmonary disease, were excluded. No patient had clinical signs of an infection at the time of their examination. The mean interval between transplantation and the CT examination was 11 months (range 5–65 months). CT examinations and lung function tests were performed within 24 hours of each other.

### CT Data Acquisition

CT examinations were performed at full inspiration (insp) and full expiration (exp) using a 64-row MDCT scanner (Lightspeed VCT, GE Healthcare, Milwaukee, WI, USA), and no intravenous contrast medium was used.

The CT data were aquired using 120 kV, 100 mAs, a rotation time of 0.8 s, and a pitch of 0.984; the slice collimation during acquisition was 1.25 mm. Data reconstruction yielded 1.25-mm slices with an interval of 1 mm using a “standard” reconstruction kernel (soft-tissue). The field of view (FOV) was adapted according to the size of the patient’s lung. No separate reconstructions of the right or left lung were performed.

Patients were instructed to hold their breath during full inspiration and expiration, respectively, during the CT data acquisition. CT data were acquired under spirometric control in order to gain information regarding the vital capacity at the time of the examination and a stable breathhold phase during data acquisition after deep inspiration and expiration, respectively.

Inspiratory and expiratory scans were performed using the same scan protocol. The mean CTDI was 10.1 mGy for both the inspiratory and expiratory CT (range: 3.36–21.9 mGy, SD: 5.08 mGy) and the mean DLPw amounted to 384.3 mGy×cm for the inspiratory and 385.8 mGy×cm for the expiratory scan (range: 117.0–890.5 mGy×cm, SD: 199.5 mGy×cm).

### Lung Function Tests

Pulmonary function tests (PFT) were performed using body plethysmography (BodyScope N, Ganshorn Medizin Electronic GmbH, Münnerstadt/Niderlauer, Germany) and the measured values were related to the predicted values calculated according to Quanjier et al. [27]. Spirometry was performed according to the guidelines provided by the American Thoracic Society and the European Respiratory Society [28].

### Quantification of the Airway Wall Parameters

For automatic quantification of the airway wall thickness (WT), the lumen diameter (LD), and the wall area percentage (WA%), dedicated software (MEVIS airway examiner, Fraunhofer MEVIS Bremen, Germany) was used [20]. The WA% was calculated as the ratio of the bronchial wall area and the total area (sum of the bronchial wall area and the bronchial lumen area). The difference of the WT between expiration and inspiration (WTdiff) was then calculated separately for each bronchial generation. After fully automatic segmentation of the bronchial tree, a central pathway through the bronchial structures was calculated. The WT and WA% were automatically measured for each cross-sectional image perpendicular to the central pathway after segmentation of the wall contours. Areas not appropriate for measurement, i.e. branching points or areas of adherence of the bronchial wall and vascular structures, were automatically excluded from the measurements. The software highlighted the automatic delineation of the bronchial wall (Figure 2), thus allowing for visual control of the computed segmentation. In cases of incorrect identification of the bronchial wall, the corresponding slice could be manually excluded from the quantitative analysis as a manual segmentation correction was not possible. For the quantitative analysis, two bronchial branches were chosen, the posterior basal segmental bronchus (B10) of the right lung and the apicoposterior segmental bronchus (B01) of the left lung as, therefore, considered data from the upper and lower parts of the lung and from both lungs, could thus be included. We chose the right lower lobe to avoid potential interference of the measurements with the motion artifacts caused by cardiac pulsation in the left lower lobe.

**Figure 2:** Bronchial wall measurements using the MeVis Airway Examiner. A three-dimensional display of the tracheobronchial tree (B) allowed the selection of the bronchus that should be evaluated (yellow border). For visualization, curved mulitplanar reformation (D) and cross-sectional images perpendicular to the central path, were used (C) and with the viewing direction along the bronchial path. The original dataset is shown in (A) and the selected bronchus is tagged with a cross-line. The location for measurements of the bronchial wall was visualized with a yellow line for the inner and a red line for the outer borderline of the bronchial wall (C).

The path of a bronchus was divided in anatomical generations following the anatomic branching from lobar, segmental to subsegmental, and sub-sub-segmental generations and with each ramification defining the beginning of a new generation. Bronchi up to the 7^th^ generation were consistently identified in all scans. More peripheral bronchi up to the 10^th^ generation could not be identified in all scans and were thus only considered if automatic segmentation was successful on both inspiration and expiration. Only bronchial generations with at least 10 valid measurements were included in the analysis. To ensure that the measurement positions were in identical bronchial generations during inspiration and expiration, all images and measurement locations were visually controlled by L.P. und S.D. The WT difference during inspiration and expiration was then calculated. The mean WT of each bronchial generation of inspiration and expiration scans was thereby assessed.

### Measurement of Lung Volumes

Lung volumes on inspiration and expiration were measured using MEVIS Pulmo (Fraunhofer MEVIS Bremen, Germany) [29].

### Statistical Analysis

Statistical tests were performed using PASW statistics (ver. 18.0, SPSS Inc., Chicago, IL, USA, 2006). The Kolmogorov-Smirnov-test was used to test normal data distribution. The correlation of PFT with the CT measurements obtained bronchus-wise for WT and WA% on inspiration and expiration CT scans, was tested using Pearson’s rank correlation coefficient.

The airway wall parameters of stable lung transplant recipients were compared with those of patients with manifested BOS using the independent samples t-test. The WA% and WT measured on inspiration were compared to the expiratory values using the paired samples t-test. To further evaluate the influence of lung volume on bronchial wall measurements, we performed a univariate analysis of variance for The WT and WA% on inspiration and expiration with the lung volume as a covariate comparing patients with and without BOS. This test compares both patient groups considering the depency of the lung volume on measurements.

## Results

### Airway Dimensions

In the entire study group (without and with BOS), the WT was measured in 2,978 bronchial generations (1,784 on inspiratory scans and 1,194 on expiratory scans) and the WA% in 2,975 bronchial generations (1,786 on inspiratory scans and 1,189 on expiratory scans). The WT difference on inspiration and expiration could be calculated for 1,079 bronchial generations.

The WT continuously decreased when moving from the central (mean WT insp 1^st^ generation: 1.76 mm) to the peripheral bronchial generations (mean WT insp 8^th^ generation: 0.81 mm) (table 2). For all generations the mean WT and mean WA% were significantly greater (paired t-test) on expiration than on inspiration (p<0.001, Table 2, Figure 3) except for the WT in the 1^st^ generation (main bronchus).

**Figure 3:** Cross-sectional images perpendicular to the central path of a segmental bronchus (B10) in a patient without (a+b) and one with BOS (c+d) during inspiration (a+c) and expiration (b+d). Differences in the WT between inspiration and expiration are visually apparent in both patients.

**Table 2:** Mean airway wall parameters during inspiration (insp) and expiration (exp) according to the bronchial generation (1 is central, 8 is peripheral).

Generation	WT insp	WT exp	p	WA% insp	WA% exp	p	WTdiff
**1**	1.76 (0.32)	1.82 (0.38)	0.166	36.53 (5.83)	41.22 (9.52)	<0.001	0.12
**2**	1.49 (0.33)	1.70 (0.34)	<0.001	39.27 (8.02)	47.07 (10.57)	<0.001	0.25
**3**	1.38 (0.34)	1.62 (0.40)	<0.001	41.87 (8.68)	50.72 (11.13)	<0.001	0.33
**4**	1.27 (0.40)	1.49 (0.43)	<0.001	43.69 (8.27)	52.85 (11.54)	<0.001	0.26
**5**	1.14 (0.43)	1.37 (0.44)	<0.001	42.86 (8.18)	52.39 (11.59)	<0.001	0.22
**6**	1.09 (0.42)	1.32 (0.41)	<0.001	42.12 (8.65)	53.98 (10.19)	<0.001	0.24
**7**	1.00 (0.31)	1.26 (0.34)	<0.001	41.47 (6.91)	56.03 (10.04)	<0.001	0.27
**8**	0.81 (0.20)	1.11 (0.31)	<0.001	36.91 (7.10)	53.66 (8.76)	<0.001	0.30

The WT (mm) and WA% (%) were significantly different between inspiration and expiration (the standard deviation values are in parentheses).

### Pulmonary Function Tests

The pulmonary function test values are shown in Table 3.

**Table 3:** Results (mean values) of the pulmonary function tests for the entire study population and subdivided according to male/female patients and those with/without BOS.

	Mean	Min	Max	standard deviation	Mean male	Mean female	Mean without BOS	Mean with BOS
	total	total	total					
**VC (ml)**	3390	1030	5780	1107	3791	2829	3575	2610
**VC/pred**	0.81	0.22	1.24	0.22	0.79	0.85	0.87	0.57
**PEF (l/min)**	6.42	1.01	11.7	2.1	7.08	5.48	1.61	3.96
**PEF/pred**	0.8	0.14	1.19	0.23	0.79	0.81	0.87	0.46
**MEF25 (l/min)**	1.39	0.12	6.01	0.97	1.57	1.14	1.61	0.42
**MEF25/pred**	0.73	0.05	2.79	0.49	0.78	0.68	0.85	0.21
**MEF50 (l/min)**	3.12	0.16	9.55	1.75	3.52	2.57	3.58	1.07
**MEF50/pred**	0.68	0.03	1.61	0.36	0.73	0.63	0.78	0.22
**MEF25–75 (l/min)**	2.74	0.15	8.7	1.55	3.08	2.27	3.17	0.85
**MEF25–75/pred**	0.71	0.04	0.83	0.39	0.76	0.66	0.83	0.21
**FEV1 (ml)**	2481	330	4690	930	2754	2115	2754	1298
**FEV1/pred**	0.74	0.09	1.33	0.25	0.74	0.74	0.82	0.36
**% of best FEV1**	84	23	102	19	84	85	92	45
**Tiffeneau**	0.73	0.26	1	0.16	0.72	0.74	0.78	0.48

### Correlation of the Airway Wall Parameters and the Lung Function Parameters

The Kolmogorov-Smirnov-test showed that the datasets for bronchial wall measurement for each bronchial generation were distributed normally. Pearson’s rank correlation coefficient was used to test the correlation between the CT morphologic and lung function parameters.

The analysis did not find any correlation of the overall WT, WA%, and WTdiff with lung function parameters determined on inspiration and expiration (Tables 4 and 5).

**Table 4:** Pearson’s rank correlation coefficient for the WT and WA% on inspiration for all bronchial generations (1^st^−10^th^).

	VC	VC/pred	PEF	PEF/pred	MEF25	MEF25/pred	MEF50	MEF50/pred	MEF25–75	MEF25–75/pred	FEV1	FEV1/pred	% best FEV1	Tiffeneau
WT generation 1	0.117	0.048	0.075	0.034	−0.021	−0.023	−0.001	−0.016	0.002	<−0.001	0.081	0.048	0.061	−0.039
WT generation 2	−0.041	−0.166	−0.086	−0.176	−0.173	−0,159	−0.110	−0.117	−0.151	−0.141	−0.121	−0.180	0.103	−0.148
WT generation 3	−0.028	−0.207	−0.071	−0.206	−0.174	−0.187	0.117	−0.150	−0.152	−0.184	−0.125	−0.213	0.103	−0.159
WT generation 4	0.009	−0.135	0.004	−0.099	−0.148	−0.157	−0.018	−0.044	−0.066	−0.091	−0.052	−0.143	0.126	−0.072
WT generation 5	0.040	−0.069	<−0.001	−0.086	−0.093	−0.084	−0.006	−0.018	−0.025	−0.027	−0.003	−0.054	0.151	−0.085
WT generation 6	0.112	−0.073	0.016	−0.127	−0.098	−0.116	−0.051	−0.092	−0.062	−0.082	0.026	−0.091	0.024	−0.150
WT generation 7	0.196	−0.059	0.098	−0.129	−0.044	−0.109	0.009	−0.070	0.010	−0.055	0.135	−0.060	0.282	−0.102
WT generation 8	−0.353	−0.358	−0.348	−0.348	−0.223	−0.147	−0.102	−0.061	−0.165	−0.084	−0.331	−0.276	0.288	−0.060
WA% generation 1	−0.061	0.062	<−0.001	0.105	−0.036	0.001	−0.011	0.022	−0.029	0.004	−0.009	0.084	0.052	0.106
WA% generation 2	−0.162	−0.170	−0.209	−0.213	−0.235	−0.205	−0.205	−0.191	−0.233	−0.203	−0.230	−0.214	0.072	−0.178
WA% generation 3	−0.256	−0.281	−0.289	−0.320	−0.246	−0.220	−0.241	−0.231	−0.257	−0.251	−0.320	−0.318	0.091	−0.192
WA% generation 4	−0.276	−0.347	−0.263	−0.314	−0.287	−0.276	−0.229	−0.229	−0.260	−0.267	−0.345	−0.378	0.205	−0.189
WA% generation 5	−0.224	−0.291	−0.260	−0.322	−0.252	−0.236	−0.216	−0,214	−0.226	−0.226	−0.280	−0.300	0.191	−0.195
WA% generation 6	−0.221	−0.336	−0.309	−0.406	−0.254	−0.243	−0.270	−0.275	−0.270	−0.267	−0.298	−0.350	0.095	−0.259
WA% generation 7	−0.073	−0.277	−0.051	−0.225	−0.162	−0.199	−0.110	−0.154	−0.117	−0.169	−0.087	−0.214	0.318	−0.008
WA% generation 8	−0.509	−0.487	−0.321	−0.319	−0.190	−0.116	−0.147	−0.101	−0.145	−0.086	−0.404	−0.327	0.480	0.111

For the airway parameters no statistically significant correlation with the lung function parameters was found (all r<0.5 except PEF and the ratio of PEF/PEF_predicted_ with WT insp in generation 10).

**Table 5:** Pearson’s rank correlation coefficient for the WT and WA% on expiration for all bronchial generations and subdivided into bronchial generations (1^st^8^th^).

	VC	VC/pred	PEF	PEF/pred	MEF25	MEF25/pred	MEF50	MEF50/pred	MEF25–75	MEF25–75/pred	FEV1	FEV1/pred	% best FEV1	Tiffeneau
WT generation 1	0.005	−0.115	−0.005	−0.079	0.099	0.073	0.069	0.039	0.062	0.037	0.016	−0.044	0.011	−0.044
WT generation 2	0.043	−0.056	−0.301	−0.110	−0.112	−0.154	−0.050	−0.078	−0.057	−0.087	−0.022	−0.092	−0.019	−0.135
WT generation 3	0.068	−0.018	0.039	−0.019	−0.031	−0.048	0.026	0.016	0.001	−0.019	0.008	−0.043	0.049	−0.075
WT generation 4	0.105	0.009	0.097	0.027	−0.118	−0.144	−0.015	−0.040	−0.046	0.097	0.022	−0.049	0.081	−0.102
WT generation 5	0.018	−0.032	−0.087	−0.137	−0.216	−0.219	−0.120	−0.126	−0.150	−0.150	−0.086	−0.127	−0.051	−0.201
WT generation 6	0.076	−0.011	0.051	−0.007	−0.039	−0.075	0.054	0.028	0.027	0.052	0.034	−0.032	−0.076	−0.027
WT generation 7	0.187	0.082	0.076	−0.011	−0.011	−0.072	0.080	0.031	0.062	0.023	0.126	0.028	0.065	−0.087
WT generation 8	0.209	0.255	0.021	0.052	−0.069	−0.097	0.009	−0.007	−0.022	−0.025	0.100	0.121	−0.215	−0.053
WA% generation 1	−0.068	−0.029	−0.118	−0.076	−0.149	−0.111	−0.153	−0.123	−0.180	−0.143	−0.126	−0.065	0.020	−0.043
WA% generation 2	−0.116	−0.052	−0.143	−0.102	−0.302	−0.304	−0.284	−0.282	−0.302	−0.290	−0.199	−0.171	−0.015	−0.165
WA% generation 3	−0.113	−0.073	−0.146	−0.131	−0.220	−0.200	−0.183	−0.167	−0.216	−0.197	−0.172	−0.140	0.004	−0.127
WA% generation 4	−0.092	−0.073	−0.169	−0.164	−0.325	−0.320	−0.329	−0,321	−0.347	−0.336	−0.189	−0.181	0.079	−0.178
WA% generation 5	−0.112	−0.047	−0.241	−0.213	−0.381	−0.371	−0.371	−0.361	−0.400	−0.383	−0.235	−0.199	−0.045	−0.229
WA% generation 6	−0.120	−0.079	−0.192	−0.173	−0.289	−0.286	−0.266	−0.254	−0.287	−0.279	−0.208	−0.182	−0.100	−0.165
WA% generation 7	0.029	0.067	−0.113	−0.115	−0.238	−0.235	−0.205	−0.205	−0.225	−0.206	−0.061	−0.035	−0.008	−0.121
WA% generation 8	0.011	0.075	−0.076	−0.035	−0.227	−0.235	0.121	−0.120	−0.159	−0.153	−0.084	−0.029	−0.176	−0.061

No statistically significant correlation with the lung function parameters was found between morphometric analysis of the airway parameters on expiration and PFT.

For the airway parameters no statistically significant correlation with the lung function parameters could be found except for Peak expiratory flow (PEF) and the ratio of PEF/PEF_predicted_ with WT insp in the 10^th^ generation, which we regard as coincidential (Tables 4 and 5).

### Comparison of the Airway Wall Parameters in Patients with and without BOS

Twenty-five examinations were performed in patients with clinically identified BOS, of which 15 were BOS stage 3. In these 25 examinations, the WT and WA% were measured in 469 bronchial generations. These were compared with the WT and WA% measurements of 2,509 and 2,506 bronchial generations, respectively, in patients without clinical evidence of BOS.

The mean WT on inspiration was slightly higher in patients with BOS than in those without BOS (Table 6), although the difference was not statistically significant. The WT on expiration did not differ significantly with and without BOS, and in the peripheral bronchial generations the WT was slightly higher in patients without BOS. The WA% on inspiration in patients with BOS differed significantly from the measurements seen in stable lung transplant recipients in most bronchial generations (Table 6). The LD is increased in the peripheral bronchial generations in patients with BOS compared to patients without BOS, and thus indicating the development of bronchiectasis (Table 7) although without statistical sgnificance.

**Table 6:** Mean WT (mm) and WA% (%) in patients without and with BOS (the standard deviation values are in parentheses).

Generation	WT insp	WT insp	WT insp	WT exsp	WT exsp	WT exsp	WA% insp	WA% insp	WA%	WA% exsp	WA% exsp	WA%
		BOS	p		BOS	p		BOS	insp		BOS	exsp
									p			p
**1**	1.86	1.79	0.356	1.8	1.82	0.808	40.03	35.71	0.003	41.23	41.98	0.751
	(0.42)	(0.39)		(0.34)	(0.46)		(8.41)	(7.08)		(8.56)	(12.04)	
**2**	1.53	1.62	0.167	1.69	1.67	0.793	40.58	44.32	0.024	47.43	47.67	0.916
	(0.37)	(0.30)		(0.33)	(0.46)		(8.32)	(9.14)		(10.51)	(11.47)	
**3**	1.39	1.52	0.056	1.63	1.66	0.756	42.57	45.27	0.182	51.29	52.65	0.529
	(0.39)	(0.42)		(0.37)	(0.53)		(8.78)	(11.67)		(10.65)	(12.38)	
**4**	1.25	1.37	0.089	1.51	1.47	0.620	43.64	48.35	0.008	52.85	54	0.627
	(0.41)	(0.44)		(0.41)	(0.54)		(8.02)	(10.32)		(11.76)	(9.80)	
**5**	1.11	1.25	0.074	1.36	1.44	0.380	42.83	47.13	0.018	51.84	56.22	0.092
	(0.43)	(0.49)		(0.43)	(0.48)		(8.00)	(10.53)		(11.76)	(10.94)	
**6**	0.98	1.04	0.496	1.31	1.3	0.947	40.95	45.34	0.064	53.58	56.76	0.236
	(0.45)	(0.44)		(0.41)	(0.35)		(8.70)	(12.39)		(10.28)	(9.46)	
**7**	0.87	1	0.107	1.26	1.21	0.719	39.33	43.96	0.015	56.24	53.91	0.561
	(0.31)	(0.34)		(0.34)	(0.36)		(7.85)	(7.08)		(10.12)	(8.81)	
**8**	0.72	0.9	0.122	1.13	0.95	0.261	35.57	42.49	0.063	54.24	49.46	0.313
	(0.22)	(0.44)		(0.31)	(0.26)		(7.25)	(13.01)		(9.12)	(3.86)	

Significant differences were found for the WA% on inspiration.

**Table 7:** The mean lumen diameter (LD) in millimeter in patients with and without BOS.

Generation	LD insp	LD insp	LD insp
		BOS	p
**1**	12.9	12.7	0.799
	(2.82)	(1.97)	
**2**	10.1	9.9	0.848
	(2.08)	(2.32)	
**3**	8.8	8.9	0.929
	(2.30)	(2.31)	
**4**	7.5	7.3	0.719
	(1.98)	(2.53)	
**5**	6.7	6.2	0.440
	(1.85	(2.51)	
**6**	6.2	6.5	0.750
	(1.89)	(2.12)	
**7**	5.8	7.6	0.017
	(1.37)	(1.20)	
**8**	5.6	6.4	0.265
	(1.15)	(1.60)	

The LD is increased in the peripheral bronchial generations in patients with BOS indicating the development of bronchiectasis. although it failed to demonstrate statistical significance with the exception of 7^th^ generation which we regard as an accidental occurrence (the standard deviation values are in parentheses).

The WT and WA% on expiration as well as the WTdiff did not differ significantly in the two patient groups. The WT and WA% were significantly larger on expiration than on inspiration in patients with and without BOS (table 2).

Lung volumes could be measured on 140 of 141 CT examinations. The lung volumes on inspiration in patients with BOS (mean: 4,903 ml) were lower than in patients without BOS (mean: 5,302 ml), although the difference was not significant (p = 0.173). The lung volumes on expiration in patients with BOS (mean: 3,178 ml) were significantly larger than those seen in patients without BOS (mean: 2,495 ml, p = 0.001). The lung volume difference between inspiration and expiration was significantly less in patients with BOS (mean: 1,840 ml) than in patients without BOS (mean: 2,815 ml, p<0.001) (table 8).

**Table 8:** The mean lung volumes during inspiration (lung vol insp) and expiration (lung vol exp) and the difference between inspiration and expiration (lung vol diff) in patients with and without BOS.

	without BOS (ml)	with BOS (ml)	p-value
**lung vol insp**	5302 (1340)	4903 (1013)	0.173
**lung vol exp**	2495 (832)	3178 (968)	0.001
**lung vol diff**	2815 (964)	1840 (863)	<0.001

The mean lung volume on expiration (lung vol exp) and the difference between the mean lung volume on inspiration and expiration (lung vol diff) differed significantly (the standard deviation values are in parentheses).

The univariate analysis of variance for the WA% revealed a significant influence of lung volume for the WA%. The univariate analysis of variance for the WT and WA%, comparing patients with and without the lung volume as a covariate, revealed a significant difference of the WA% on inspiration in either case (Table 9). Both the presence of BOS and the different lung volume had significant influence on measurements of the WA% on inspiration. The WT on inspiration and expiration and the WA% on expiration did not show a significant difference in either group with and without using the lung volume as a cofactor.

**Table 9:** Level of significance for univariate analysis of variance for the WT (mm) and WA% on inspiration and expiration and corrected for lung volume comparing patients with and without BOS.

	influence of lung volume				corrected for lung volume			
Generation	WA% insp	WT insp	WA% exp	WT exp	WA% insp	WT insp	WA% exp	WT exp
**1**	0.096	0.024	0.554	0.057	0.002	0.527	0.692	0.841
**2**	0.045	0.498	0.003	0.271	0.076	0.177	0.415	0.889
**3**	<0.001	0.461	0.002	0.463	0.361	0.052	0.233	0.633
**4**	<0.001	0.370	0.113	0.398	0.007	0.087	0.636	0.469
**5**	0.001	0.572	0.136	0.172	0.035	0.076	0.114	0.377
**6**	0.013	0.231	<0.001	0.011	0.100	0.556	0.073	0.609
**7**	0.026	0.525	0.165	0.206	0.018	0.102	0.788	0.933
**8**	0.007	0.916	0.007	0.263	0.009	0.015	0.478	0.337

There was a significant influence in the lung volume on the WA% (columns 1–4) and also a significant difference in the WA% on inspiration in patients with and without BOS even if considering the differing lung volumes as cofactor (colums 5–8).

However, the variability of bronchial wall measurements was high and the values for the WA% on inspiration in patients with and without BOS, overlapped considerably (Figure 4).

**Figure 4:** Boxplot showing the average WA% in patients with and without BOS, according to bronchial generations in inspiration. Despite significant differences in the WA% between patients with and those without BOS, there is a substantial overlap in both patient groups.

## Discussion

In our study, only the WA% on inspiration differed significantly in patients with and without BOS. Therefore, WA% seems to be more suitable for diagnosing BOS than the WT. However, there was a high variability of the measurements due primarily to variable underlying lung volumes which minimize the value of WA% for establishing a diagnosis of BOS based on the imaging findings in individual patients.

CT morphologic parameters and lung function parameters have been found to have statistically significant correlations for a number of airway diseases that differ with respect to the type and anatomic location of their underlying pathology as well as the distribution within the lung. For example, a moderate correlation between the CT airway morphology (WA or LA) and lung function (FEV_1_) could be found in patients with COPD [19], [20], those with CF [21], and in patients with asthma [22], [23].

BOS primarily affects the small airways with diameters<2 mm [1] that cannot be resolved on CT. This raises the question whether bronchial wall measurements of CT data are at all a useful tool for the assessment of BOS. However, previous studies have shown that wall thickening of visually discernible bronchi, i.e. more central bronchial segments, is usually found in patients with BOS [9]. It has also been shown that in patients with COPD the bronchial wall dimensions in relatively large airways, as measured on CT, correlate with those of small airways measured histologically [30]. These reports regarding the meaning of airway CT morphology in other airways diseases [19], [21], [22] and the fact that bronchial wall thickening is also included as a separate criterion in the CT scoring system for BOS [31] motivated us to perform this study. The goals of our prospective study set-up were: a) to assess bronchial wall dimensions in lung transplant patients without clinical symptoms of BOS; and b) to compare those dimensions with the bronchial wall dimensions of patients with BOS.

In our study we used validated software to detect the WT and the WA% [20]. This software is based on the closed-form solution [19] which is optimized to reduce overestimation of the WT in small airways and is, therefore, specifically suited for lung transplant patients with pathologically small airways. We used the standard reconstruction kernel rather than the sharper lung kernel as it has been shown that this kernel provides more robust measurements [32]. All measurements were carried out automatically and were thus independent of any user interaction or the CT window settings. Multiple measurements per bronchial generation, in our study at least 10, provided reliable data to also allow for analysis of individual bronchial segments. As there are non-anatomical branching points and smaller branches that might be missed by the program, the measuring points did not necessarily conform to the bronchial generations [19]. To ensure that the measurement locations were identical on inspiration and expiration, all images and measurements were visually checked and “outliers” were eliminated to further increase the accuracy of the quantification.

In our study, there was no correlation of the bronchial wall measurements and the lung function tests performed in lung transplant recipients with and without BOS. The WT on inspiration was slightly higher in patients with BOS than in patients without BOS. This was expected as bronchial wall thickening has been noted in patients with BOS [9], and bronchial wall thickening is used in the CT scoring systems for BOS [31]. However, the difference of the WT on inspiration did not reach statistical significance in those patients with and without BOS. This might be due to the high, dependency of airway measurements on the degree of inspiration, as already shown for the lumen area [33]. This is further supported by the fact that the WT and the WA% were significantly larger on expiration than on inspiration. Regarding the lung volumes that were lower on inspiration and significantly higher on expiration in patients with BOS compared to those without BOS, this might indicate that the influence of the lung volume on measurement of the WT is higher than the presence of BOS. In contrast to the WT, the WA% on inspiration was found to be significantly higher in most bronchial generations in patients with BOS compared to that seen in stable lung transplant patients (Table 5). Therefore, the WA% appears to be a better predictor of BOS than the WT. The WA% is calculated as the ratio of the bronchial wall area and the total area (sum of bronchial wall area and bronchial lumen area). The development of bronchiectasis in patients with BOS leads to a decrease in the WA% (the total area is the denominator and increases in bronchiectasis), whereas bronchial wall thickening results in an increase in the WA% (the wall area is the numerator). As the WA% is higher in patients with BOS, the increase in wall area seems to be more relevant than the development of bronchiectasis. However, the WA% also varied according to the lung volume and showed significantly higher values on expiration than on inspiration. On expiration, the WT increases due to shrinking of the bronchial lumen diameter. The WA% also increases on expiration as the total area (denominator) decreases due to reduction of the bronchial lumen although the wall area (numerator) generally remains the same (the reduced diameter is compensated for by an increased WT). The lung volumes in patients with BOS were non-significantly lower on inspiration and significantly greater on expiration than those in patients without BOS, probably due to obstructive changes. This suggests that the smaller inspiratory lung volumes in patients with BOS contribute to the significant increase of the WA%. This agrees with the study of Zach et al. who showed that the WA% is strongly related to the total lung capacity [34]. In order to be able to eliminate the influence of the lung volume on the difference of the WA% in patients with and those without BOS, we performed a univariate analysis of variance considering the lung volume as a covariate. We could, therefore, confirm the significant influence of the lung volume on the WA%, although we also found significant differences for the WA% on inspiration for the two patient groups after correcting for the influence of the lung volume. These results suggest that the WA% on inspiration is an indicator of both the presence of BOS and the differences in lung volume. However, the inter- and intravariability of the bronchial wall measurements was high in our study. This is not surprising as it is known from pathology studies that BOS shows a very nonuniform anatomic distribution [7]. This makes it necessary to acquire a large number of bronchial wall measurements. Whether bronchial wall measurements alone will be sufficient to diagnose BOS cannot be determined on the basis of our rather small study group. Given the overlap of measurements in patients with and those without BOS, it seems to be more likely at that point that bronchial wall measurements might be a useful adjunct combined with other CT morphologic features such as the presence and amount of air trapping noted on CT. In the future, it will be worthwhile to evaluate whether longitudinal bronchial wall measurements in individuals after lung transplantation are sufficient to document the progression of bronchial wall thickening in patients with increasing symptoms of BOS and vice versa for those undergoing therapy. Furthermore, it might be interesting to evaluate whether a correcting factor for lung volume can be calculated for bronchial wall measurements as this might help to eliminate the influence of lung volume on measurements. Moreover, it may also be worthwhile to differentiate between patients with the fibrotic and inflammatory phenotypes of BOS.

Our study has a number of limitations. All bronchial wall measurements were performed using one type of software tool. Although the underlying algorithm of this software was thoroughly tested and well-established [19], [20], different software tools might yield different results for quantification. Secondly, the number of patients with clinically manifested BOS was much smaller than those without BOS. Also, the number of patients with different severity of BOS stages was too small to allow for a meaningful analysis of the patient subgroups. It is already known that BOS does not occur uniformly or equally affect all bronchi in the lungs. However, in order to provide an objective and standardized method for measurements with high reproducibility we specified the target bronchi prior to the evaluation and did not individually select the target bronchi. In this study we focused on analysis of the bronchial wall measurements and did not include other CT morphological findings such as air trapping. Inclusion of those criteria and the use of airway wall measurements in longitudinal studies will be the foci of future studies.

## Conclusion

WA% on inspiration was significantly greater in patients with than in those without BOS. However, WA% measurements were significantly dependent on lung volume and showed a high variability, thus not allowing the sole use of bronchial wall measurements to differentiate patients with from those without BOS.

## References

[1] Al-GithmiI, BatawilN, ShigemuraN, HsinM, LeeTW, et al (2006) Bronchiolitis obliterans following lung transplantation. Eur J Cardiothorac Surg 30: 846–51.1705528310.1016/j.ejcts.2006.09.027

[2] BoehlerA, KestenS, WederW, SpeichR (1998) Bronchiolitis obliterans after lung transplantation: a review. Chest 114: 1411–26.982402310.1378/chest.114.5.1411

[3] ArcasoySM, KotloffRM (1999) Lung transplantation. N Engl J Med 340: 1081–91.1019423910.1056/NEJM199904083401406

[4] ToddJL, PalmerSM (2011) Bronchiolitis obliterans syndrome. Chest 140: 502–8.2181352910.1378/chest.10-2838

[5] CooperJD, BillinghamM, EganT, HertzMI, HigenbottamT, et al (1993) A working formulation for the standardization of nomenclature for clinical staging of chronic dysfunction in lung allografts: International Society for Heart and Lung Transplantation. J Heart Lung Transplant 12: 713–6.8241207

[6] EstenneM, MaurerJR, BoehlerA, EganJJ, FrostA, et al (2002) Bronchiolitis obliterans syndrome 2001: an update of the diagnostic criteria. J Heart Lung Transplant 21: 297–310.1189751710.1016/s1053-2498(02)00398-4

[7] ChamberlainD, MaurerJ, ChaparroC, IdolorL (1994) Evaluation of transbronchial lung biopsy specimens in the diagnosis of bronchiolitis obliterans after lung transplantation. J Heart Lung Transplant 13: 963–71.7865530

[8] BankierAA, Van MuylemA, KnoopC, EstenneM, GevenoisPA (2001) Bronchiolitis obliterans syndrome in heart-lung transplant recipients: diagnosis with expiratory CT. Radiology 218: 533–9.1116117510.1148/radiology.218.2.r01fe09533

[9] MorrishWF, HermanSJ, WeisbrodGL, ChamberlainDW (1991) Bronchiolitis obliterans after lung transplantation: findings at chest radiography and high-resolution CT. The Toronto Lung Transplant Group. Radiology 179: 487–90.201429710.1148/radiology.179.2.2014297

[10] KonenE, GutierrezC, ChaparroC, MurrayCP, ChungT, et al (2003) Bronchiolitis obliterans syndrome in lung transplant recipients: can thin-section CT findings predict disease before its clinical appearance? Radiology 231: 467–73.10.1148/radiol.231203056315128992

[11] NgYL, PaulN, PatsiosD, WalshamA, ChungTB, et al (2009) Imaging of lung transplantation: review. AJR Am J Roentgenol 192: S1–13.1923428410.2214/AJR.07.7061

[12] MillerWTJr, KotloffRM, BlumenthalNP, AronchickJM, GefterWB, et al (2001) Utility of high resolution computed tomography in predicting bronchiolitis obliterans syndrome following lung transplantation: preliminary findings. J Thorac Imaging Apr 16(2): 76–80.10.1097/00005382-200104000-0000211292208

[13] BerstadAE, AaløkkenTM, KolbenstvedtA, BjørtuftO (2006) Performance of long-term CT monitoring in diagnosing bronchiolitis obliterans after lung transplantation. Eur J Radiol 58: 124–31.1638746510.1016/j.ejrad.2005.11.013

[14] CoxsonHO (2008) Quantitative computed tomography assessement of airway wall dimensions: current status and potential applications for phenotyping chronic obstructive pulmonary disease. Proc Am Thorac Soc. 15 5(9): 940–5.10.1513/pats.200806-057QCPMC272010819056721

[15] BrilletPY, FetitaCI, Beigelman-AubryC, SaragagliaA, PerchetD, et al (2007) Quantification of bronchial dimensions at MDCT using dedicated software. Eur Radiol 17(6): 1483–9.1711516010.1007/s00330-006-0496-7

[16] NakanoY, MullerNL, KingGG, NiimiA, KallogerSE, et al (2002) Quantitative assessment of airway remodeling using high-resolution CT. Chest 122: 271S–5S.12475796

[17] NakanoY, WhittallKP, KallogerSE, CoxsonHO, FlintJ, et al (2002) Development and validation of human airway analysis algorithm using multidetector row CT. Proc SPIE 4683: 460–469.

[18] ReinhardtJM, D'SouzaND, HoffmanEA (1997) Accurate measurement of intrathoracic airways. IEEE Trans Med Imaging 16: 820–7.953358210.1109/42.650878

[19] WeinheimerO, AchenbachT, BletzC, DuberC, KauczorHU, et al (2008) About objective 3-d analysis of airway geometry in computerized tomography. IEEE Trans Med Imaging 27: 64–74.1827006310.1109/TMI.2007.902798

[20] SchmidtM, KuhnigkJM, KrassS, OwsijewitschM, de HoopB, et al (2010) Reproducibility of airway wall thickness measurements. PROC SPIE doi:10.1117/12.844453

[21] AchenbachT, WeinheimerO, BiedermannA, SchmittS, FreudensteinD, et al (2008) MDCT assessment of airway wall thickness in COPD patients using a new method: correlations with pulmonary function tests. Eur Radiol 18: 2731–8.1864199310.1007/s00330-008-1089-4

[22] HasegawaM, NasuharaY, OnoderaY, MakitaH, NagaiK, et al (2006) Airflow limitation and airway dimensions in chronic obstructive pulmonary disease. Am J Respir Crit Care Med 173(12): 1309–15.1655669510.1164/rccm.200601-037OC

[23] MontaudonM, BergerP, Cangini-SacherA, de DietrichG, Tunon-de-LaraJM, et al (2007) Bronchial measurement with three-dimensional quantitative thin-section CT in patients with cystic fibrosis. Radiology 242: 573–81.1717939910.1148/radiol.2422060030

[24] MontaudonM, LederlinM, ReichS, BequeretH, Tunon-de-LaraJM, et al (2009) Bronchial measurements in patients with asthma: comparison of quantitative thin-section CT findings with those in healthy subjects and correlation with pathologic findings. Radiology 253: 844–53.1978921910.1148/radiol.2533090303

[25] ChaeEJ, KimTB, ChoYS, ParkCS, SeoJB, et al (2011) Airway Measurement for Airway Remodeling Defined by Post-Bronchodilator FEV1/FVC in Asthma: Investigation Using Inspiration-Expiration Computed Tomography. Allergy Asthma Immunol Res 3: 111–7.2146125010.4168/aair.2011.3.2.111PMC3062789

[26] GottliebJ, SzangoliesJ, KoehnleinT, GolponH, SimonA, et al (2008) Long-term azithromycin for bronchiolitis obliterans syndrome after lung transplantation. Transplantation 15 85(1): 36–41.10.1097/01.tp.0000295981.84633.bc18192909

[27] QuanjerPH, TammelingGJ, CotesJE, PedersenOF, PeslinR, et al (1993) Lung volumes and forced ventilatory flows. Report Working Party Standardization of Lung Function Tests, European Community for Steel and Coal. Official Statement of the European Respiratory Society. Eur Respir J 16: 5–40.8499054

[28] MillerMR, HankinsonJ, BrusascoV, BurgosF, CasaburiR, et al (2005) Standardization of spirometry. Eur Respir J 26: 319.1605588210.1183/09031936.05.00034805

[29] KuhnigkJM, DickenV, ZidowitzS, BornemannL, KuemmerlenB, et al (2005) New Tools for Computer Assistance in Thoracic CT - Part I: Functional analysis of lungs, lung lobes, and bronchopulmonary segments. RadioGraphics 25: 525–536.1579806810.1148/rg.252045070

[30] NakanoY, WongJC, de JongPA, BuzatuL, NagaoT, et al (2005) The prediction of small airway dimensions using computed tomography. Am J Respir Crit Care Med 15 171: 142–6.10.1164/rccm.200407-874OC15516531

[31] de JongPA, DoddJD, CoxsonHO, Storness-BlissC, ParéPD, et al (2006) Bronchiolitis obliterans following lung transplantation: early detection using computed tomographic scanning. Thorax 61: 799–804.1667017010.1136/thx.2005.053249PMC2117084

[32] KimN, SeoJB, SongKS, ChaeEJ, KangSH (2008) Semi-automatic measurement of the airway dimension by computed tomography using the full-width-half-maximum method: a study on the measurement accuracy according to the CT parameters and size of the airway. Korean J Radiol 9: 226–35.1852522510.3348/kjr.2008.9.3.226PMC2627250

[33] BakkerME, StolkJ, ReiberJH, StoelBC (2012) Influence of inspiration level on bronchial lumen measurements with computed tomography. Respir Med 106(5): 677–86.2215424710.1016/j.rmed.2011.11.013

[34] ZachJA, NewellJDJr, SchroederJ, MurphyJR, Curran-EverettD, et al (2012) on behalf of the COPDGene Investigators (2012) Quantitative Computed Tomography of the Lungs and Airways in Healthy Nonsmoking Adults. Invest Radiol 47: 596–602.2283631010.1097/RLI.0b013e318262292ePMC3703944

